This article has been retracted.

# Global Increase in Breast Cancer Incidence: Risk Factors and Preventive Measures

**DOI:** 10.1155/2022/9605439

**Published:** 2022-04-18

**Authors:** Dharambir Kashyap, Deeksha Pal, Riya Sharma, Vivek Kumar Garg, Neelam Goel, Deepika Koundal, Atef Zaguia, Shubham Koundal, Assaye Belay

**Affiliations:** ^1^Department of Histopathology, Postgraduate Institute of Medical Education and Research, Chandigarh 160012, India; ^2^Department of Translational and Regenerative Medicine, Postgraduate Institute of Medical Education and Research, Chandigarh 160012, India; ^3^Department of Pulmonary Medicine, Postgraduate Institute of Medical Education and Research, Chandigarh 160012, India; ^4^Department of Medical Laboratory Technology, University Institute of Applied Health Sciences, Chandigarh University (Gharuan), Mohali 140313, India; ^5^Department of Information Technology, University Institute of Engineering & Technology, Panjab University, Chandigarh 160014, India; ^6^Department of Systemics, School of Computer Science, University of Petroleum & Energy Studies, Dehradun, India; ^7^Department of computer science, College of Computers and Information Technology, Taif University, P.O. BOX 11099, Taif 21944, Saudi Arabia; ^8^Department of Statistics, Mizan-Tepi University, Ethiopia

## Abstract

Breast cancer is a global cause for concern owing to its high incidence around the world. The alarming increase in breast cancer cases emphasizes the management of disease at multiple levels. The management should start from the beginning that includes stringent cancer screening or cancer registry to effective diagnostic and treatment strategies. Breast cancer is highly heterogeneous at morphology as well as molecular levels and needs different therapeutic regimens based on the molecular subtype. Breast cancer patients with respective subtype have different clinical outcome prognoses. Breast cancer heterogeneity emphasizes the advanced molecular testing that will help on-time diagnosis and improved survival. Emerging fields such as liquid biopsy and artificial intelligence would help to under the complexity of breast cancer disease and decide the therapeutic regimen that helps in breast cancer management. In this review, we have discussed various risk factors and advanced technology available for breast cancer diagnosis to combat the worst breast cancer status and areas that need to be focused for the better management of breast cancer.

## 1. Introduction

Breast cancer is a leading health concern among women due to its high mortality and morbidity rate The five-year survival rate in metastatic breast cancer is less than 30%, even with adjuvant chemotherapy [1]. Recent GLOBOCAN 2018 data produced by the IARC (International Agency for Research on Cancer) from 185 countries reported 2.3 million new cases (11.7%) of breast cancer and a mortality rate of 6.9% [2]. Breast cancer incidence is more common in high-income countries (571/100 000) than in low-income counties (95/10 000), reflecting the association with globalization. Breast cancer is usually called a group of disease (>100) due to the presence of various biological subtypes reflecting distinct molecular profile and clinicopathological features [2, 3] (Figure 1). Other than histological subtypes, gene expression profiling has classified breast cancer into different molecular subtypes, i.e., receptor-positive (Luminal A, Luminal B, Normal like, and HER-2 (Human epidermal growth factor receptor) 2 positive ) and receptor-negative (TNBC (Triple negative breast cancer)) or Basal like) (Figure 1) [4–6]. Lehmann et al. further identified the different groups named in TNBC subtypes Basal like-1, Basal like-2, Immunomodulatory, Mesenchymal, Mesenchymal Stem Cell like, and Luminal Androgen depending upon expression of distinct genes [7]. The overall collective data identified that these breast cancer subtypes have different histopathological and clinical behaviors and are associated with different age groups and ethnicities [4, 8, 9], such as TNBC and HER-2 positive subtypes which are notably common in younger and premenopausal women, more prevalent in African-American and Asian women, exhibiting more metastatic potential with high relapse rate [10–15]. In developed countries, modified lifestyle, delayed age for marriage, late first child, late-night work schedule, and hormonal replacement therapy are the major risk factors for breast cancer development [16, 17]. In developing countries, the main reasons for high breast cancer incidence and mortality are lack of proper awareness or knowledge of the disease, inappropriate screening programs, delayed diagnosis, and insufficient medical facilities [18, 19]. There are multiple therapies available for breast cancer treatment including surgery, radiotherapy, chemotherapy, endotherapy, and immunotherapy [20, 21]. Despite the availability of these therapies, breast cancer incidence and mortality remain high [22, 23]. In the way of resolving this problem, multiple omics studies identified intra and intertumor heterogeneity in breast cancer which is the leading cause for relapse or resistance to treatment therapies [23–26]. Further, scientific researchers and clinicians are continuously developing or improving present knowledge and technologies to explore tumor heterogeneity in breast cancer. Improvement or advancement in sequencing tools, such as next-generation sequencing, single-cell sequencing, spatial gene expression profiling, and bioinformatics support, is providing significant support on tumor heterogeneity [27–29]. Also, several authorized agencies are screening the women at high breast cancer risk to reduce the breast cancer incidence. Despite these facilities, a number of new breast cancer cases are still increasing. The main reason is the lack of accurate information and loop in utilizing the availability of these facilities. In addition, currently, the COVID-19 pandemic around the world caused health system or screening programs closures, delay in diagnosis or treatment availability, and increases in advanced-stage diagnoses and mortality [30–35]. The present review article will summarize the current status of breast cancer morbidity and mortality, major risk factors behind, and possible strategies for the prevention of breast cancer risk.

## 2. Risk Factors for Breast Cancer

Epidemiological studies correlated different factors for breast cancer risk development or progression (Table 1) [36, 37]. Risk factors including late age for marriage, first childbirth, and menopause are strongly associated with disease development (Figure 2) [38–40]. A study estimated the risk of 7.0% (95% confidence interval: 5.2, 9.1) in women who married at age 30 or older, relative to women who married at a younger age (~20 year), whereas the corresponding risk was 1.4% (95% confidence interval: 1.1, 1.8) when marriage age was less than 30 but the first childbirth age is 30 or more [41]. Late age at marriage and childbirth leads to lack of breast tissue differentiation, more exposure to nonestrogenic mutagens, and genotoxicity by estrogen [42]. Menopause after 50 years of age puts the women at prolonged estrogen exposure [43, 44]. A meta-analysis study observed that early pregnancy and longer breastfeeding duration reduce ER (Estrogen receptor) positive and ER negative breast cancer risk [45, 46]. Similarly, unbalanced diet intake is another factor associated with breast cancer risk. Study estimated that women on nonvegetarian and high animal fat diet had more chance of breast cancer development than women on vegetarian diet [47–49]. Further, poor physical activity also correlated to breast cancer risk. In a case-control study conducted in the south Indian population determined that women engaged in household activities had low breast cancer risk compared to women not involved in household activities [50, 51]. In addition, obesity (high waist-to-hip ratio) is another strong risk factor for breast cancer in postmenopausal women and also associated with poor disease outcome in women of all ages [52–54]. In the United States, about 18% of premenopausal women have elevated BMI and are at high breast cancer development risk [55]. It was observed that postmenopausal women with ≥5.0 BMI (Body Mass Index) and ≥90 cm abdominal circumference were more likely to develop breast cancer [56, 57]. It results from the activity and accumulation of polycyclic aromatic hydrocarbons (PAH) in breast fat tissue. In the breast fat tissue, PAH interacts with the cellular estrogen receptor to enhance the risk of development of breast cancer [58]. Besides, another study noted that obese women with breast cancer have worse disease-free and overall survival than nonobese women with breast cancer. [52]. Moreover, a study found that moderate alcohol consumption of >35-44 grams/day increases 46% (95% CI = 1.33-1.61) risk for breast cancer [59–61]. In breast tissue, higher dose of alcohol is metabolized to acetaldehyde by alcohol dehydrogenase enzyme. Accumulated acetaldehyde can bind to proteins and DNA and interferes with the antioxidative defense system, DNA synthesis, and repair system by downregulating BRCA1 (BReast CAncer gene 1) [62–65]. Hormonal contraception formulations contain lower doses of estrogen, but its use for long time can also put the women at high breast cancer risk (RR=1.20; 95% CI=1.14-1.26) [66].

## 3. Epidemiology

In 2018, approximately 6.8 million women across the world were living with breast cancer. But the information in cancer registries is incomplete, it is not documented that how many women have metastatic spread and are now cancer free, as only incidence or mortality is being registered in cancer registries [67, 68]. Wide variations in education levels, economic status, environmental conditions, food habits, lifestyle factors, and other cultural practices cause difference in the incidence of breast cancer across the world. Globalization and growing economy may further exacerbate breast cancer incidence in developing (64% to 95) and developed (32% to 56%) countries by 2040 [69, 70]. In urban India, high breast cancer incidence reported was in the age group of 40–49 years, while in rural areas, it was between 65 and 69 years [71]. A study from northern India population documented that 26% of patients detected with breast cancer were less than 35 years of age [72]. Difference in the eating patterns such as consumption of tobacco (smoked versus smokeless tobacco), alcohol (spirits versus wines), and nonvegetarian diet (high amount red meat vs. low amount of red meat) also accounts for variation in the breast cancer incidence [37].

### 3.1. International Breast Cancer Burden

Recently, the GLOBOCAN 2020 data by the IARC (International Agency for Research on Cancer) reported worst breast cancer incidence and prevalence in 185 countries (Figure 3) [69]. Breast cancer is the leading most commonly diagnosed cancer with a total of 2.3 million new cases (11.7%) of breast cancer [69]. Further, as per estimated the number of new breast cancer cases and deaths in US were 0.28 million and 0.04 million, respectively [73]. As an estimation, one in 4 women has breast cancer, and one in 8 women died due to breast cancer disease [69]. According to the American Cancer Society, global cancer burden would be 28.4 million cases by 2040, which is ~47% raise compared to 2020 cancer burden [74]. Women in older age have high breast cancer incidence. In 2018, 6,45,000 vs. 1·4 million breast cancer cases and 130,000 vs. 490,000 deaths were reported in the premenopausal and postmenopausal group, respectively [69]. It is reported that countries with high human development index (HDI) has the highest premenopausal (30.6/100,000) and postmenopausal (253.6/100,000) breast cancer incidence [75], while countries with low and medium HDI had the lowest premenopausal (8.5/100,000) and postmenopausal mortality (53.3/100,000) [76]. Insufficiency to approach for early diagnosis and effective treatment remains a crucial factor for higher breast cancer mortality in developing countries [75].

### 3.2. National Breast Cancer Burden

Breast cancer remains the fast-growing cancer in India after crossing cervical cancer. National Cancer Registry Program in 2018 estimated ~1,62,468 new breast cancer cases and ~87,090 deaths due to breast cancer in India [77, 78]. Annual percentage change in the incidence of breast cancer ranged from 0.46% to 2.56% which crossed cervical cancer in 2012. According to a survey carried out by the ICMR (Indian Council of Medical Research) New Delhi, breast cancer incidence has almost doubled from 1982 to 2005 [79]. It is noted that breast cancer is more common in the younger population and has poor prognosis in India compared to the Western world [80]. A local study found 52% of breast cancer-suffering women were between 40 and 49 years of age and a significant number were below 30 years of age [81]. The survival rate in India is very poor due to the detection of disease at an advanced disease stage. Usually, 60% of women present with TMN (tumor size, metastasis, and lymph node) stage III with 80% lymph node positivity and only 1.4% presents with stage I [82]. The mean breast cancer tumor size reported in India is 3.56cm and ranged from <2cm in 18.2%, 2-5cm in 65.1%, and >5cm in 16.7% cases [78, 81], whereas in USA, 64% of patients present with local disease, 28% with regional spread, and 6% with distant spread of disease. The late presentation of the disease is influenced by socioeconomic status, level of education, marital status, and residence [72]. The age-adjusted incidence rates for breast cancer (AAR) in different cities of India including Delhi, Chennai, Bangalore, Mumbai, and Kolkata are 41%, 38%, 34.4%, 33.6%, and 25.5% cases per 100,000 population [15, 83]. Considering breast cancer subtypes distribution, TNBC is the more common and highly prevalent subtype in Indian women and accounts about 20-43% of total breast cancer patients [15]. A meta-analysis study found a higher prevalence of TNBC subtype in India compared to in Western populations. Different risk factors, primarily including lifestyle, deprivation status, obesity, family history, high mitotic indices, and BRCA1 mutations, might be associated with increased incidence of TNBC in the Indian population [84]. HER-2 positive subtype is also observed to be highly prevalent in young Indian women. On the contrary Luminal A subtype in younger Indian women is lowest compared to other races [15]. This alarming scenario emphasizes a multidisciplinary approach for breast cancer management, including extensive breast cancer screening and awareness programs and easily approachable medical facilities to all the women in urban and rural India. A detailed strategy is needed for the hour to reduce breast cancer incidence and mortality.

## 4. Different Available Approaches to Control Breast Cancer

An extensive breast cancer information program, to create awareness among the people regarding risk factors and incidence of breast cancer, is of utmost importance. In addition, screening programs and diagnostic tests are essential for early detection to reduce the burden of breast cancer incidence and mortality [85].

### 4.1. Molecular Testing

Breast cancer is a genetic disease that results due to change in the genomic structure [86]. Genetic alterations in tumor suppressor and oncogenic genes transform breast epithelial cell to malignant phenotype [87]. These genetic alterations also affect the behavior of breast cancer including response to therapy and clinical outcome. Significant advancements in molecular techniques have made breast cancer diagnosis and treatment decision more convenient. Currently, conventional histopathological methods along with molecular testing are integrated to classify molecular subtypes of breast cancer more accurately. Molecular diagnosis has shown an unprecedented impact on breast cancer management. Molecular testing helps in identifying a certain set of genes as biomarkers that might help to predict prognosis of the disease and efficacy of the treatment. Different assays are now available to check the expression of various genes involved in different breast cancer progressions [5]. For example, PAM50 (Prediction Analysis of Microarray 50) an FDA-approved multigene kits to understand better breast tumors and prognostication in ER-positive, HER-2-negative, lymph node-negative, and >5cm tumor size breast cancers [88–90]. Microarray-based PAM 50 consists of 50 genes to test the breast tumor samples for the risk of distant recurrence for postmenopausal women within 10 years of diagnosis. If PAM50 score comes out to be high, it shows a fairly high risk of metastasis [91]. It is advisable to plan treatment strategy accordingly. ONCOTYPE DX is another assay kit, a predictive model of breast cancer testing [92–94]. It is a 21-gene expression assay that calculates the risk of breast cancer relapse. ONCOTYPE DX provides the information using tumor section and predicts locoregional disease recurrence that helps in making decision about the radiotherapy for postmenopausal women with ER/PR positive and node positive breast cancer [95, 96]. Further, ENDOPREDICT (EndoPredict®) is RNA-based 12 gene (8 cancer-related genes, 3 reference genes, and one control gene to check DNA contamination) assay kit [97, 98]. It aids in providing information of DCIS (ductal carcinoma in situ) risk and disease recurrence. Patients with ER-positive, HER-2-negative, stage I/II, and lymph node negative status are eligible for EndoPredict testing [99, 100]. In addition, MammaPrint was designed by the Netherlands Cancer Institute (NKI) in Amsterdam and was approved by the FDA in 2007. MammaPrint is a microarray-based commercialized assay that measures the 70 gene expressions and can predict the metastasis in ER/PR+/-, stage I or stage II, >5 cm, and three or fewer lymph nodes early-stage breast cancer [101]. It predicts relapse of stage 1 or stage II hormone receptor positive and hormone receptor negative tumors within 10 years of diagnosis. In IMPACT trial, clinically high-risk and 70-gene signature low-risk patients, there was a 60% reduction in treatment recommendations [102]. Also, urokinase-type plasminogen activator, a proteolytic enzyme that breakdowns the extracellular matrix and helps in metastasis, is another prognostic calculator assay kit [103, 104]. Plasminogen is converted onto its active form plasmin by tissue-type (tPA) and the urokinase-type (uPA) activators. It is evident from trials reported that elevated uPA and PAI-1 levels predict poor clinical outcome [105, 106]. Similarly, Breast Cancer Index test predicts the cancer relapse after 5 to 10 years of diagnosis in hormone receptor positive and node negative breast cancer patients. Therefore, molecular diagnostic assays are integrated as a part of breast cancer management as they estimate risk of metastasis, tumor recurrence, and therapy response. Outcome of the result helps the clinician to decide the time frame for the hormonal therapy in a patient.

### 4.2. Next Generation Sequencing

Improvement in traditional sequencing technologies with extraordinary depth reads counts and analysis of entire genome in a single experiment, which is the unprecedented achievement in molecular biology [107–110]. The massive parallel and deep sequencing technologies called Next Generation Sequencing (NGS) have revolutionized the genomic research [111]. Next generation sequencing is a cost-effective method that provides complete genome information using a multigene panel in a single set of experiment. This high throughput technique provides information of gene variants, gene alteration, point mutations, gene fusion, and copy number variation [112]. This advanced sequencing technique in the diagnosis of breast cancer has been widely accepted throughout the world as it is contributing to patient-specific therapies. Various reasons for the popularity of NGS in diagnostics are attributed to several added advantages that include ultrahigh throughput, scalability, and speed. Reversible dye terminator method (Illumina) and semiconductor ion proton (ThermoFisher Scientific), SMRT PacBio, and Nanopore (Oxford) enable the identification of different somatic and germ line genetic aberrations (SNP, CNV, Indel, translocation, and gene expression), protein expressions, and epigenetic alterations with high accuracy and sensitivity. RNA sequencing (RNA-Seq) can quantify the copy number of different cellular RNA species in different tissues and can discover the novel or splice site mRNA variants [113]. In addition, NGS is also in practice to study the genome wide epigenomic modifications such as histone modification, DNA methylation, and DNA-protein interaction [114]. Similarly, Nanopore DNA sequencing device developed by the Oxford Nanopore Technologies is a simple experimental process that analyze DNA strand directly as the molecule passes through tiny pore suspended in membrane [115]. The device works on change in the current as the different combinations of G, A, T, and C nucleotides pass through the pore made up of protein sets [116]. This cost-effective approach has advantages to read label-free, ultralong (10^4^ to 10^6^ bases) sequence, rapid processing, real-time result display, and generate high-throughput data even with low material. Phenotypic and molecular heterogeneity in tumor is mainly responsible for therapy failure and therapy resistance [117, 118]. Understanding and decoding of tumor heterogeneity would help to improve the survival rate in breast cancer patients. In this context, single-cell sequencing with template switch method has advantages to decode the tumor heterogeneity over the bulk sequencing data [119–121]. Further, mapping the spatial organization of an intact tissue section using spatially resolved high-resolution transcriptomics deciphered tumor heterogeneity [122]. Spatial molecular imaging technologies, including sequential Fluorescence in Situ Hybridization (seq FISH) [123], Fluorescent In Situ Sequencing (FISSEQ) [124], GeoMx [125], Slide-seq [126], STARmap [127], High-Definition Spatial Transcriptomics (HDST) [128], and Multiplexed Error-Robust Fluorescence In Situ Hybridization (MERFISH), enable the analysis thousands of RNAs and proteins from single cells with subcellular resolution in morphologically intact tissue samples [122]. The spatial molecular imaging combines the power of high-plex profiling with high-resolution imaging and allows researchers to visualize and quantify targeted protein and gene expression on tissue slices [129]. Further, there are many online repository databases containing the information of all three omics on breast cancer. Databases such as TCGA (The Cancer Genome Atlas) [130, 131], GEO (Gene Expression Omnibus) [132, 133], and METABRIC (Molecular Taxonomy of Breast Cancer International Consortium) have genetic, transcriptomic, protein expression, and epigenetic information derived from a significant number of breast cancer patients. These databases also have clinicopathological features of breast cancer patients and can be used for meta-analysis.

### 4.3. Liquid Biopsy

Tumor biopsy is a gold standard method to determine the disease pathology at cellular level for diagnosis [134]. Spatial and temporal heterogeneity exists in cancer and limits the advantages of solid tumor biopsy procedures [135, 136]. Repeat invasive procedures are not advisable in clinical setting. All these drawbacks can be overcome by liquid biopsy due to ease of sample extraction and cost effectiveness and can be repeated to monitor the disease progression. Due to effectiveness of liquid biopsy, it seems as a future of diagnosis [137]. Recent advancements of DNA sequencing and molecular diagnosis have promoted circulating tumor DNA (ctDNA) as a marker for liquid biopsy [138–140]. Currently, FDA-approved test kits such as Cobas EGFR Mutation Test V_2_ for the treatment monitoring of non-small-cell lung carcinoma, Epi proColon test for the detection of colorectal cancer, and Guardant360 CDx and FoundationOne Liquid CDx provide clinically relevant information [141–143]. Similarly, CellSearch is another FDA-approved kit for the assessment of CTC (circulating tumor cell) in metastasis breast, colon, and prostate cancer [144, 145]. A study screened ESR1 (p.Leu536Arg, p.Tyr537Ser, p.Tyr537Asn, p.Tyr537Cys, and p.Asp538Gly) in cell-free plasma of 171 breast cancer patients using ultrahigh sensitivity multiple digital droplet PCR [146]. In a clinical trial, the early-stage TNBC patients received neoadjuvant chemotherapy, which measured ctDNA that was negatively correlated with overall survival, disease-free survival, and distant disease-free survival [147]. Thus, liquid biopsy sequencing analysis is a promising option to extract the information of somatic mutational landscape in a less invasive procedure.

### 4.4. Genetic Testing

Robust research work identified and associated the several genetic aberrations in different genes with disease onset and clinical outcome [148]. Genetic testing, supported by advancement in genetic sequencing techniques and bioinformatics tools, allows the efficient detection of germline mutations in breast cancer patients. Genetic testing in breast cancer has substantial implications for cancer prevention, early detection, and treatment for patients and their relatives (Table 2) [149]. Since the last three decades, the germline genetic testing for inherited breast cancer risk prediction has evolved substantially [150]. The most frequently mutated and/or amplified genes reported in the tumor cells for early breast cancer detection are TP53 (41% of tumors), PIK3CA (Phosphatidylinositol-4,5-Bisphosphate 3-Kinase Catalytic Subunit Alpha) (30%), MYC (20%), PTEN (Phosphatase and Tensin Homolog deleted on Chromosome 10) (16%), CCND1 (Cyclin D1) (16%), ERBB2 (Erb-B2 Receptor Tyrosine Kinase 2) (13%), FGFR1 (Fibroblast growth factor receptor 1) (11%), and GATA3 (10%). Several genes with germline mutations have been identified which are related with hereditary breast cancer [151]. Genes including BRCA1/2, CDH1 (Cadherin 1), PALB2 (Partner And Localizer Of BRCA2), PTEN, STK11 (Serine/threonine kinase 11), and TP53 are significantly associated with hereditary breast cancer [152–156]. Information of carrier for these gene mutations in the family can help to manage hereditary disease in the family. Mutation in BRCA1, BRCA2, and PALB2 is associated with the development of breast cancer in 1 out of 10 cases. Mutation in BRCA1 and BRCA2 is distributed in all population of the world; BRCA1 and BRCA2 are responsible of 45% hereditary breast cancer cases [157–160]. It is mandatory to look for BRCA1 and BRCA2 mutations and understand the specific pathological features of BRCA-associated tumors and specific molecular cascade involved in it [161, 162]. Other genes such as ATM (Ataxia telangiectasia mutated), CHEK2 (Checkpoint kinase 2), BARD1 (BRCA1-Associated RING Domain 1), BRIP1 (BRCA1-Interacting Protein 1), NBN (Nibrin), RAD51C (RAD51 Paralog C), RAD51D, and NF1 (Neurofibromin 1) with pathogenic mutations have twofold to fourfold increased risk for breast cancer [163]. Family history, race, and ethnicity affect the prevalence of germline mutations and the associated risk therefore should be considered during genetic testing or risk assessment estimating. Breast cancers are usually caused cumulatively by multiple and low penetrant mutations. Certain gene mutations are subtype-specific, i.e., Luminal A tumors have a high prevalence of PIK3CA mutations (49%) and basal-like tumors have high prevalence of TP53 mutations (84%) [130, 151, 164]. Mutated BRCA gene is usually found in TNBC subtypes, whereas CHEK2 and ATM mutations are commonly occurred in ER-positive breast cancer subtypes. [165–167]. Few studies gave guidelines for genetic testing. In 2019, the American Society of Breast Surgeons (ASBrS) proposed germline genetic testing for all breast cancer patients to increase the identification of pathological variant carriers [168]. Over the guidelines of the NCCN (National Comprehensive Cancer Network) and ASBrS, a Mayo Clinic study in 2020 proposed a hybrid approach for germ genetic testing for all diagnosed breast cancer patients with 65 years age using the NCCN criteria for older patients [149]. Keeping ≤60 or ≤65 years of age for universal testing has detected more pathological variants (11.9% and 15.7% respectively) in comparison with using the NCCN criteria [169]. Despite the benefits of genetic testing, a significant number of breast cancer patients never undergo for genetic testing. The lack of facility, patient awareness, cost, and an inadequate genetic counseling workforce are the main barriers. Racial and ethnic disparities in genetic testing also exist, and this can influence evidence-based cancer surveillance, prevention, and cancer treatment for these groups. Integrated and updated guidelines, BRCA testing for identification of BRCA carriers would help for both preventive and therapeutic purposes [163, 170].

### 4.5. Artificial Intelligence

In addition to the wet lab work, computer-based algorithm can also help to understand the disease etiology [171]. Artificial intelligence (AL) is an emerging area which aims at designing computer structures that simulate human intelligence. Machine learning (ML) comes under AI that design advance algorithms in helping to understand the disease behavior [172]. Accumulated data evidenced that ML can improve the breast cancer diagnosis and help predict the prognosis. For example, Osareh et al. [173] differentiated the benign from malignant mass with the help of digitalized images of Fine Needle Aspirate biopsy samples [174]. Similarly, few authors integrated and interpreted digital histopathological images with DL technique to identify histological subtypes and grade in breast cancer samples [175]. Further, algorithms have been designed to explore the inter and intratumor heterogeneity [176, 177] and cellular subsets such as neutrophils, macrophages, and fibroblast in breast cancer TME. Machine learning algorithms have also been developed for immunohistochemical subtyping and measurement of ER/PR [178], HER-2 positive, and Ki-67 antibody positive cells [179, 180]. Moreover, with the help of AI, Whitney et al. [173] predicted relapse risk ER+ breast cancer patients. In more advanced way, AI approach can be used to determine the correlation of proliferation and cell cycle markers for personalized therapy [181]. Therefore, abovementioned data promising that AI in the future can provide larger information may be used for the diagnosis and treatment of breast cancer.

## 5. Approaches to Implement

### 5.1. Cancer Registry

A cancer registry is a surveillance process that collects the data of cancer incidence, mortality, diagnosis, and treatment. It is required for policy making to implement the efforts required to control cancer incidence and identify the areas to focus for cancer prevention [85, 182, 183]. Presently, most of the cancer registries focused on collection of data at two time points, i.e., at the time of incidence (diagnosis) and at death (mortality). For the better strategies to combat worse breast cancer situations, the cases should be thoroughly followed for survival estimation and treatment response. All this information will be of help in drawing the effectiveness of diagnosis, therapeutics, and overall cancer services in a particular area. In India, cancer registry was started in 1960s, and presently, it includes 36 PBCRs (Population-based cancer registry) and 236 HBCRs (Hospital-based cancer registry) [85, 182]. In India, cancer registry programs are not effective due to skewed distribution of cancer hospitals and PBCRs and mostly data in urban centric data. Moreover, cancer registry is not mandatory in India. Now, cancer registry programs in India are being revised. Innovative online programs and cancer atlas are being included so as to streamline cancer registration.

### 5.2. Screening Program

Establishing primary prevention programs for breast cancer remains a challenge. Population-wide breast cancer screening programs aim at reducing breast cancer mortality through early detection and effective treatment. Effective implementation of population-based screening programs is the need of the hour and could be a way of improving the health outcomes of women [184]. Mammography-based screening is highly beneficial and recommended for early detection of the breast tumor [185]. In the United Kingdom (UK), women between the age of 50 and 71 years are invited for breast cancer screening every three years [186]. Mammography can detect the presence of any abnormality; therefore, extensive screening program results in more chances of survival. In India, breast cancer screening program is still in its infancy and there is no well-organized breast cancer screening program at present. It results in late detection at advance stage which is the main reason behind the high mortality rate in India [187]. As per the National Family Health Survey, 2015–2016 (NFHS-4), breast cancer morbidity and mortality is highest in India [184]. In India, cancer incidence is high in 40-60 age group; therefore, screening should be more focused on this age group [81]. Mammography is not easily affordable in India and clinical breast examination is cost-effective. The Ministry of Health and Family Welfare, India, has recommended CBE every 5 years for women between 30 and 65 years of age group by primary health-care worker [82]. The WHO advocates mammography-based screening once in every 2 years for 50 to 69 years of age group. [188, 189]. The American Cancer Society recommends annual screening from 40 to 44 years age group of women [190]. Sometimes mammographic screening can lead to false-positive results; to improve this situation, a risk stratified should be utilized using risk prediction models [191, 192]. Magnetic resonance imaging (MRI) and mammography together is recommended for women with BRCA1 and/or BRCA2 mutations [193–195]. Mammography randomized controlled trials have shown that population screening significantly reduces mortality from breast cancer by 20% [196, 197].

## 6. Bench to Bedside

Molecular technologies have discovered different types of biomarkers for diagnosis, prognosis, drug resistance, and therapeutic implications. These biomarkers may help in resolving the problem of drug resistance in breast cancer treatment. Change in the DNA methylation pattern is associated with the carcinogenesis. For instance, more than 90% of breast cancer patients showed methylated promotor of adenomatous polyposis coli (APC) and retinoic acid receptors-2 (RARb2) gene [198]. Utilizing a human methylation in a BeadChip DNA study by Yang et al., hypomethylation of S100 calcium-binding protein P (S100P) and hyalurono glucosaminidase 2 (HYAL2) was observed to be correlated with adolescent breast cancer patients [199, 200]. Noncoding RNAs such as circular RNAs (circRNAs) and microRNAs (miRNAs) have been identified over the years showing promising noninvasive diagnostic and prognostic performance of the breast cancer. The miR-221, miR-21, and miR-145 in the blood serum or plasma of breast cancer individuals have shown higher diagnostic susceptibility than CEA and CA 15–3 for all stages of cancer [201–203]. Iorio et al. in 2005 identified deregulated miRNAs (mir-125b, mir-145, mir-21, and mir-155) in breast cancer patients [204]. Also, Blenkiron et al. in 2007 discovered 133 miRNAs in human breast tissue and breast tumor tissue. About 1/8th part of the human genome is transcribed into circRNAs [205]. Due to the circular structure and nonterminal end, these RNA molecules are most stable in all kinds of body fluids [206, 207]. Lu et al. reported upregulated hsa circ 103110, hsa circ104689, and hsa circ104821 [AUC value of 0.63 (0.52–0.74), 0.61 (0.50–0.73), and 0.60 (0.49–0.71), respectively] and downregulated hsa circ006054, hsa circ100219, and hsa circ406697 [AUC value of 0.71 (0.61–0.81), 0.78 (0.69–0.88), and 0.64 (0.52–0.75), respectively] in the breast cancer patients [208]. As per the published literature, all these omics biomarker have clinical potential and need to be explored further for clinical value.

## 7. Conclusion

Epidemiological data of breast cancer accumulated so far sought the severity of the disease. Sensitive, specific, easily available, and cost-effective diagnostic and therapeutic approaches are urgently required for the reduction of breast cancer incidence and prevalence. Several strategies are described in the present review articles which are being used around continents. Diagnostic or predictive biomarkers cannot be used commonly in all the regions due to their varied values based on the ethnicity. Effectiveness of preventive and screening programs also depends on the economic condition of the country. Therefore, good validation of the biomarkers is required to decide the region specific cut off values. In addition, a great data for all three omics is accumulated at the research levels only. To bring this information into the clinic, we need a large-scale validation. Workout of all these issues would reduce the incidence and prevalence of breast cancer.

## 8. Future Perspective

Great data suggest that each breast cancer patients has distinct genetic, transcriptional, and epigenetic profile. Different studies explored the breast cancer heterogeneity using genetic (mutation) and genomic information (gene expression). For example, Ciriello et al. used copy number and mutational landscape data from multiple studies and classified the Luminal A breast cancer subtype into different groups (i.e., mixed, copy number high, chromosome 8 associated, copy number quiet, and 1q/16q) [209]. This heterogeneity at phenotypic and molecular in breast cancer reduces the treatment efficacy and hence clinical outcome. Genome profiling of individual patient can explore the molecular heterogeneity and would be useful for personalized medicine. Further improvement in the next generation technologies including further high accuracy, sensitivity, and low-cost for availability to each patient is required. Although, discovery of DNA, RNA, protein- and epigenetic-based diagnostic, and therapeutic biomarker would improve the breast cancer understanding, the non-reproducibility of these markers between the patients in intra and intercontinents limits their use. The most effective prevention approach for breast cancer is the awareness of disease. There should be organized awareness and screening programs for breast cancer at different levels. Every woman should know their breast and should teach about breast cancer and self-screening. Women with high breast cancer risk should take extrapreventive measures including counseling and clinical consultation.

## Figures and Tables

**Figure 1:** Schematic representation of (a) histopathological classification, (b) molecular classification, and (c) time line showing important events during understanding of breast cancer biology.

**Figure 2:** Schematic representation of breast cancer risk factors.

**Figure 3:** Distribution of cancer incidence and mortality among different types of cancer

**Table 1:** Describing the various factors and their consequences which results in risk for breast development.

Risk factors	Consequences	Ref
Early puberty	At puberty, undifferentiated, proliferative breast cells increase rapidly and more exposure to hormonal changes increases susceptibility to mutagens	[210]
Early menarche	At menarche, breast cells tend to grow and divide increasing the risk of breast cancer	[211]
Late marriage age	Prolong exposure to estrogen hormone	[212]
Late child birth age	Lack of breast tissue differentiation and prolong exposure to estrogen hormone	[213]
Lactation failure	Lack of breast tissue differentiation, more susceptible to nonestrogenic mutagens and estrogen	[214]
Late menopause age	Late onset of breast involution and prolong exposure to estrogen and progesterone	[215]
Lack of physical activity	Reduced exposure to sex hormones due to increase the number of anovulatory cycles	[216]
High fat diet	Cholesterol activate estrogen signalling and cell proliferation	[217]
Obesity	Increased levels of inflammatory cytokines and chemokines	[52]
Alcohol consumption	Increase estrogen hormone	[218]
Smoking	Induce gene mutations such as p53 gene mutation and DNA adducts	[219]
HRT	Prolong exposure to estrogen hormone	[220]
Contraceptive	Contraceptives contain progesterone and estrogen	[221]
Family history	BRCA1/2 gene mutations	[222]
Environmental toxicants	Pollutants can disrupt endocrine signalling	[223]

**Table 2:** Genes, mutation type, and biochemical product active in breast cancer [224].

Gene	Biochemical function	Location	Mutation type	Product Type
BRCA1	DNA repair	117q21.31	Germinal/somatic	Protein coding
BRCA2	DNA repair	13q13.1	Germline/somatic	Protein coding
PIK3CA	Regulate p110 alpha	3q26.32	Somatic	Protein coding
MYC	Cellular signalling	8q24.21	Somatic	Protein coding
PTEN	Block PI3K signalling	10q23.31	Somatic/germinal	Protein coding
CCND1	Cell cycle	11q13.3	Somatic	Protein coding
ERBB2	Kinase	17q12	Somatic	Protein coding
ERBB3	Kinase	12q13.2	Somatic	Protein coding
FGFR1	Receptor	1 8p11.23	Somatic	Protein coding
FGFR2	Receptor	10q26.13	Somatic/germinal?	Protein coding
GATA3	Transcriptional factor	10p14	Somatic	Protein coding
AKT2	Kinase	19q13.2	Somatic	Protein coding
ARID1B	Chromatin remodelling	6q25,3	Somatic	Protein coding
CASP8	Apoptosis	2q33.1	Somatic/germinal?	Protein coding
CDKN1B	Cell cycle control	12p13.1	Somatic	Protein coding
MAP3K1	Kinase	5q11.2	Somatic/germinal?	Protein coding
MAP3K13	Kinase	3q27.2	Somatic	Protein coding
NCOR1	Transcriptional coregulator	17p12-p	Somatic	Protein coding
SMARCD1	Chromatin remodelling	12q13.12	Somatic	Protein coding
TBX3	Transcriptional repressor	12q24.21	Somatic	Protein coding
RB1	Cell cycle regulator	13q14.2	Somatic	protein coding
ESR1	Receptor	6q25.1-q25.2	Somatic	Protein coding
FOXA1	Transcriptional factor	14q21.1	Somatic	Protein coding
CDH1	ECM signalling	16q22.1	Somatic/germinal	Protein coding
APOBEC3B	Innate immunity	22q13.1	Somatic	Protein coding
PALB2	DNA repair	16p12.2	Germinal/somatic?	Protein coding
ATM	DNA repair	11q22.3	Germinal/somatic	Protein coding
CHEK2	DNA repair	22q12.1	Germinal/somatic	Protein coding
RAD51	Homologous recombination	15q15.1	Germinal	Protein coding
RAD51C	Homologous recombination	17q22	Germinal/somatic?	Protein coding
MSH2	DNA mismatch repair	2p21-p16	Germinal/somatic	Protein coding
BARD1	DNA repair	2q35	Germinal/somatic?	Protein coding
STK11	Kinase	19p13.3	Germinal/somatic	Protein coding
BRIP1	DNA repair	17q23.2	Germinal/somatic	Protein coding
MALAT1	Long noncoding RNA	11q13.1	Somatic	Nonprotein coding
HOTAIR	Long noncoding RNA	12q13.13	Somatic	Nonprotein coding
MEG3	Long noncoding RNA	14q32.2	Somatic	Nonprotein coding
H19	Long noncoding RNA	11p15.5	Somatic	Nonprotein coding

## Data Availability

No data were used to support this study.
